This article has been retracted.

# Clinical Effect of Nimodipine Combined with Magnesium Sulfate on Pregnancy-Induced Hypertension Syndrome

**DOI:** 10.1155/2022/7217543

**Published:** 2022-03-25

**Authors:** Ruixia Chang, Hui Miao, Ailing Cui, Lingyan Jiang, Linlin Yang, Congxiu Miao

**Affiliations:** ^1^Department of Reproduction and Genetics, Heping Hospital Affiliated to Changzhi Medical College, Changzhi 046000, China; ^2^Laboratory,Changzhi Medical College, Changzhi 046000, China; ^3^Department of Information, Heping Hospital Affiliated to Changzhi Medical College, Changzhi 046000, China

## Abstract

The incidence of pregnancy-induced hypertension in China is 9.4%, which is at a relatively high level. Its serious impact on maternal and infant health is the main reason for maternal and perinatal morbidity and mortality. There are many factors affecting pregnancy-induced hypertension. The incidence of pregnancy-induced hypertension is different due to different levels of cultural knowledge, health awareness, economic income, nutrition, and medical support. Since its etiology has not been elucidated thus far, there is no known treatment of the disease, and the main principles are spasmolysis, hypotension, expansion, and timely termination of pregnancy. Observe the effect of nimodipine combined with magnesium sulfate on serum heat shock protein 70 (HSP70) and pentamer 3 (PTX3) levels in patients with pregnancy-induced hypertension. Ninety-six patients with pregnancy-induced hypertension syndrome admitted to our hospital from May 2016 to February 2019 are selected and randomly divided into two groups according to the 1 : 1 principle, with 48 cases in each group. The single drug group is treated with magnesium sulfate, and the combined group is treated with nimodipine combined with magnesium sulfate. Changes in blood pressure, HSP70, PTX3, placental growth factor (PLGF), and vascular endothelial cell injury markers are recorded in the two groups, and adverse reactions and pregnancy outcomes are observed. After treatment, the blood pressure and levels of HSP70, PTX3, endothelin-1 (ET-1), and nitric oxide (NO) in the two groups decreased, and the level of PLGF increased. The diastolic blood pressure, systolic blood pressure, and levels of HSP70, PTX3, ET-1, and NO in the combined group are lower than those in the single drug group, and the level of PLGF is higher than that in the single drug group (*P* < 0.05). During the treatment period, the adverse reaction rate of the combined group is 6.25% compared with 8.33% of the single agent group, and the difference is not statistically significant (*P* > 0.05). Follow-up visits found that the cesarean section rate and abnormal fetal heart rate in the combined group are 16.67% and 4.17%, respectively, which are lower than 35.42% and 16.67% in the single drug group, and the difference is statistically significant (*P* < 0.05). Compared with 14.58%, 12.50%, and 2.08% in the single drug group, the neonatal asphyxia rate, premature birth rate, and stillbirth rate in the combined group are 6.25%, 4.17%, and 0.00%, respectively, and the difference is not statistically significant (*P* > 0.05). Nimodipine combined with magnesium sulfate can effectively control blood pressure in patients with pregnancy-induced hypertension, reduce vascular endothelial damage, regulate the expression of HSP70, PTX3, and PLGF, and improve pregnancy outcomes without increasing adverse reactions.

## 1. Introduction

Pregnancy-induced hypertension syndrome is a common clinical pregnancy disease that can cause adverse maternal and infant outcomes. At present, magnesium sulfate is often used for expectant treatment, but there are still some severe patients with poor curative effects. Therefore, looking for safe and effective treatments of gestational hypertension has certain practical significance. In this study, the dihydropyridine calcium antagonist nimodipine combined with magnesium sulfate is used to treat pregnancy-induced hypertension syndrome, and its efficacy is observed. HSP70, PTX3, and other indicators are detected in the laboratory to explore its mechanism of action to provide a reference for the clinical treatment of pregnancy-induced hypertension.

The pathogenesis of pregnancy-induced hypertension syndrome is complex. At present, it is believed that the expression of various inflammatory factors and growth factors is related to the occurrence and progression of pregnancy-induced hypertension syndrome [1]. Pregnancy-induced hypertension syndrome can cause symptoms such as elevated blood pressure, edema, proteinuria, dizziness, and severe preeclampsia, resulting in severe adverse consequences such as premature delivery and maternal and neonatal death [2]. Magnesium sulfate is a basic treatment for pregnancy-induced hypertension syndrome, which can relieve small vessel spasms, but its blood pressure control effect is not good, and it often needs to be combined with antihypertensive drugs [3]. Nimodipine is a dihydropyridine calcium antagonist with definite antihypertensive effects, and it can improve the peripheral circulation. Some studies have shown that nimodipine combined with magnesium sulfate has better efficacy in the treatment of pregnancy-induced hypertension syndrome [4].

Heat shock protein 70 (HSP70) has a wide range of biological effects, and it increases rapidly when the body experiences a stress response. The body of patients with pregnancy-induced hypertension is in a state of stress, and HSP70 is highly expressed [5]. Pentamer 3 (PTX3) is a downstream effector molecule of the NF-*κ*B-mediated signaling pathway, which is related to hypertension and cardiovascular disease and can protect the cardiovascular system [6]. In this study, the effects of nimodipine combined with magnesium sulfate on serum HSP70 and PTX3 levels in patients with pregnancy-induced hypertension syndrome are observed to provide a reference for clinical treatment.

## 2. Our Proposed Method

### 2.1. General Information

Ninety-six patients with pregnancy-induced hypertension syndrome admitted to our hospital from May 2016 to February 2019 are selected and randomly divided into two groups according to the 1 : 1 principle, with 48 cases in each group. The age of the single drug group is 22–35 years old, mean 28.42 ± 2.81 years old. There are 30 primiparas and 18 multiparas. The gestational age is 31–38 weeks, mean 33.96 ± 1.94 weeks, and a mean body mass index of 23.29 ± 2.11 kg/m^2^. The age of the combined group is 22–35 years old, mean 28.35 ± 2.91 years old. There are 32 primiparas and 16 multiparas. The gestational age is 31–38 weeks, mean 33.98 ± 2.03 weeks, and a mean body mass index of 23.34 ± 1.98 kg/m^2^.

The inclusion criteria are as follows: compliance with the criteria in the “Guidelines for diagnosis and treatment of hypertensive disorders in pregnancy (2012 edition)” [7]; single birth, head upright, no developmental abnormalities [8]; aged 22–35 years [9]; no other antihypertensive treatment is given before admission [10]; and patients ' informed consent. The exclusion criteria are as follows: patients with a history of diabetes, hypertension, or nephritis; patients with cardiovascular and cerebrovascular diseases or liver and kidney dysfunction; malignant tumor and mental illness; allergy to study drugs; and those who have a history of macrosomia delivery, miscarriage, or premature delivery of a huge baby. There is no significant difference in the general data between the two groups (*P* > 0.05). This study is approved by the hospital ethics committee [11, 12].

### 2.2. Method

All patients are on bed rest, fetal heart sounds are closely monitored, oxygen is inhaled intermittently, sodium intake is restricted for those with systemic edema, and symptomatic and supportive treatments such as sedation and diuresis are given. On this basis, the single drug group is given 25% magnesium sulfate injection (Harbin Pharmaceutical Group Sanjing Pharmaceutical Co., Ltd.). On the first day of treatment, 20 mL magnesium sulfate is added to 20 mL 5% glucose solution by intravenous injection. If there is no discomfort, it is increased to 35 mL from the second day. The treatment goal is maintaining blood pressure<140/90 mm Hg.

The combined group is given nimodipine injection (Biomedical Engineering Center of Hebei Medical University) combined with magnesium sulfate treatment. The dosage of magnesium sulfate is the same as above. Nimodipine (10 mg) is added to 35 mL of 5% glucose solution intravenously, and the injection is stopped when the blood pressure is maintained at approximately 140/90 mmHg. Then, oral nimodipine tablets (Hayao Group Sanjing Pharmaceutical Factory Co., Ltd.) are given 30 mg/time, 2 times/d until delivery.

### 2.3. Observation Indicators and Detection Methods

Changes in blood pressure are recorded, and adverse reactions (gastrointestinal reactions, flushing, and dry mouth) and pregnancy outcomes (cesarean section, abnormal fetal heart rate, neonatal asphyxia, premature delivery, and stillbirth) during treatment are recorded.

Five milliliters of peripheral venous blood is collected before and after 1 week of treatment, centrifuged at 4°C, speed 3000 r/min, centrifugal radius 8 cm, and time 10 min. The serum levels of placental growth factor (PLGF), heat shock protein 70 (HSP70), pentamer 3 (PTX3), endothelin-1 (ET-1), and nitric oxide (NO) are detected by enzyme-linked immunosorbent assay kits (Shanghai Enzyme-linked Biological Technology Co., Ltd.). Detection instrument is the Beckman immune analyzer. We strictly complied with the requirements of the kit instructions for operation.

SPSS 19.0 is used to process the data. The measurement indicators are described by ($\bar{x}\pm s$), the independent sample *t*-test is used for the comparison between groups, the paired *t*-test is used for the comparison within the groups, and the rate comparison is performed by the *χ*^2^ test. *P* < 0.05 is defined as statistically significant.

## 3. The Clinical Results

### 3.1. Comparison of Blood Pressure between the Two Groups

Before treatment, the blood pressure of the two groups is compared, and the difference is not statistically significant (*P* > 0.05). After treatment, the blood pressure of the two groups is lower than that before treatment, and the diastolic blood pressure and systolic blood pressure of the combined group are lower than those of the single drug group (*P* < 0.05).  Table 1 provides comparison of blood pressure in 2 groups.

### 3.2. Comparison of Two Groups of HSP70, PTX3, and PLGF

Before treatment, HSP70, PTX3, and PLGF are compared between the two groups, and the difference is not statistically significant (*P* > 0.05). After treatment, PLGF in the two groups increased, HSP70 and PTX3 decreased, and PLGF in the combined group is higher than that in the single drug group, and HSP70 and PTX3 are lower than those in the single drug group (*P* < 0.05).  Table 2 provides the comparison of HSP70, PTX3, and PLGF levels in the two groups.

### 3.3. Comparison of the Levels of Vascular Endothelial Cell Injury Markers in the Two Groups

Before treatment, vascular endothelial cell injury markers are compared between the two groups, and the difference is not statistically significant (*P* > 0.05). After treatment, ET-1 and NO in the two groups decreased compared with those before treatment, and ET-1 and NO in the combined group are lower than those in the single drug group (*P* < 0.05).  Table 3 provides comparison of the levels of vascular endothelial cell injury markers in the two groups.

### 3.4. Comparison of Adverse Reactions between the Two Groups

The adverse reactions of all patients are mild discomfort and untreated, and they recovered spontaneously. The adverse reaction rate of the combined group is 6.25%, compared with 8.33% of the single drug group, and the difference is not statistically significant (*P* > 0.05).  Table 4 provides comparison of adverse reactions between the two groups.

### 3.5. Comparison of Pregnancy Outcomes between the Two Groups

The cesarean section rate and abnormal fetal heart rate in the combined group are 16.67% and 4.17%, respectively, which are lower than 35.42% and 16.67% in the single drug group, and the difference is statistically significant (*P* < 0.05). The neonatal asphyxia rate and premature birth rate in the combined group are 6.25% and 4.17%, respectively, compared with 14.58% and 12.50% in the single drug group, and the difference is not statistically significant (*P* > 0.05). One case of stillbirth (hypoxia) occurred in the single drug group, with an incidence of 2.08%, while no stillbirth occurred in the combined group.  Table 5 provides the comparison of pregnancy outcomes between the two groups.

## 4. Data Result Analysis

Pregnancy-induced hypertension syndrome (PIH) is a late pregnancy complication that occurs more than 20 weeks after pregnancy and is the main cause of adverse pregnancy outcomes. At present, there is no specific treatment for this disease, only rest, oxygen inhalation, spasmolysis, sedation, diuretics, and other symptomatic treatments. Magnesium sulfate can inhibit the release of acetylcholine from motor nerve-muscle junctions, block the conduction of neuromuscular junctions, relieve muscle contraction, relax vascular smooth muscle, expand peripheral blood vessels, and reduce blood pressure, and it is generally the first choice for the treatment of this disease. However, its control of blood pressure is not ideal, and large doses of magnesium sulfate can also cause systemic fever, facial redness, dry mouth, and other adverse reactions.

Nimodipine is a calcium antagonist-type antihypertensive drug that can expand blood vessels, inhibit vascular smooth muscle contraction, and reduce blood pressure. At the same time, it can expand cerebral vessels and regulate peripheral circulation. It is often used in the treatment of hypertension and cerebrovascular diseases, and it has a good therapeutic effect. Since nimodipine does not cause damage to the fetus through the placental barrier, it is suitable for antihypertensive treatment of pregnant women. Studies have found that nimodipine combined with magnesium sulfate in the treatment of pregnancy-induced hypertension syndrome is beneficial to improve the overall clinical efficacy. In this study, it is found that the decrease in diastolic blood pressure and systolic blood pressure in patients treated with nimodipine combined with magnesium sulfate is better than that in patients treated with magnesium sulfate. This is consistent with the existing research reports. Magnesium sulfate can reduce blood pressure by relaxing vascular smooth muscle and expanding peripheral blood vessels, while nimodipine can relax vascular smooth muscle by inhibiting calcium influx and then produce antihypertensive effects. The two drugs have different action pathways, which can have complementary antihypertensive effects.

Many studies have shown that the stress response and vascular endothelial cell damage play an important role in the pathogenesis of pregnancy-induced hypertension syndrome. PLGF is a protective factor secreted by syncytiotrophoblast cells to promote angiogenesis and improve placental blood perfusion. HSP70 is a kind of stress protective protein that is microexpressed in normal circumstances. When the body experiences a stress response, HSP7 is highly expressed, which produces antioxidant effects, participates in regulating the body's stress state, and improves the tolerance of cells to abnormal stimuli. Pregnancy-induced hypertension can cause systemic arterial spasm, reduce the blood supply of the uterus and placenta, lead to the release of inflammatory factors, cause the formation of oxygen free radicals and oxidative stress, and increase the level of HSP70. PTX3 is a long chain molecule synthesized by granular leukocytes, endothelial cells, fibroblasts, and adipocytes. It is secreted in large quantities under the stimulation of inflammatory factors such as TNF-*α* and IL-1. It is one of the downstream effectors of the NF-*κ*B-mediated signaling pathway and has a protective effect on the cardiovascular system. Studies have found that PTX3-deficient mice have a higher risk of vascular inflammation and atherosclerosis. ET-1 and NO are specific markers of vascular endothelial cell function damage. The high expression of ET-1 and NO suggests that vasomotor dysfunction and small vessel spasms are increasing blood pressure.

In this study, the levels of HSP70, PTX3, ET-1, and NO in the two groups after treatment are lower than those before treatment, and the level of PLGF is higher than that before treatment. The levels of HSP70, PTX3, ET-1, and NO in patients treated with nimodipine combined with magnesium sulfate are lower than those in patients treated with magnesium sulfate, and the level of PLGF is higher than that in the patients treated with magnesium sulfate. This result suggests that nimodipine combined with magnesium sulfate can better reduce vascular endothelial injury and the stress response in patients with pregnancy-induced hypertension syndrome and protect the cardiovascular system.

## 5. Conclusion

In summary, nimodipine combined with magnesium sulfate can effectively control blood pressure in patients with pregnancy-induced hypertension, reduce vascular endothelial damage, regulate the expression of HSP70, PTX3, and PLGF, and improve the pregnancy outcome without increasing adverse reactions.

This study also finds that the adverse reaction rates of the two groups are similar during treatment. Follow-up showed that the cesarean section rate and abnormal fetal heart rate of nimodipine combined with magnesium sulfate are lower than those of magnesium sulfate alone. The neonatal asphyxia rate, premature delivery rate, and stillbirth rate of the two groups are similar. This is because nimodipine and nimodipine combined with magnesium sulfate can better reduce blood pressure, relieve small vessel spasms, improve the blood supply and oxygen supply of the uterus and placenta, and prevent intrauterine distress, so that the cesarean section rate and abnormal fetal heart rate can be reduced. At the present stage of obstetrics and gynecology technology, adverse pregnancy outcomes such as neonatal asphyxia, premature delivery, and stillbirth can be reduced by means of oxygen inhalation, expectant treatment, and cesarean section, which may be the reason for the similar neonatal asphyxia rate, premature delivery rate, and stillbirth rate between the two groups.

## Figures and Tables

**Table 1:** Comparison of blood pressure in 2 groups ($\bar{x}\pm s$, mmHg).

Group	Number of cases	Diastolic pressure		Systolic pressure	
		Before treatment	After treatment	Before treatment	After treatment
Single drug group	48	92.58 ± 4.67	85.25 ± 2.36^*∗*^	145.98 ± 7.84	131.25 ± 6.45^*∗*^
Joint group	48	91.97 ± 4.28	81.47 ± 2.13^*∗*#^	148.53 ± 7.55	123.02 ± 5.47^*∗*#^
*t*		0.667	8.238	1.623	6.742
*P*		0.253	≤0.001	0.054	≤0.001

*Note.* Compared with before treatment, ^*∗*^*P* < 0.05; compared with single drug group, ^#^*P* < 0.05.

**Table 2:** Comparison of HSP70, PTX3, and PLGF levels in the two groups ($\bar{x}\pm s$).

Group	Number of cases	HSP70 (ng/mL)		PTX3 (*μ*g/L)		PLGF (pg/mL)	
		Before treatment	After treatment	Before treatment	After treatment	Before treatment	After treatment
Single drug group	48	5.85 ± 1.02	2.98 ± 0.67^*∗*^	2.74 ± 0.64	2.30 ± 0.51^*∗*^	35.89 ± 5.87	158.75 ± 15.87^*∗*^
Joint group	48	5.79 ± 1.14	1.74 ± 0.55^*∗*#^	2.69 ± 0.73	1.98 ± 0.42^*∗*#^	36.11 ± 6.08	243.11 ± 26.43^*∗*#^
*t*		0.272	9.911	0.357	3.356	0.180	18.958
*P*		0.373	≤0.001	0.361	0.001	0.429	≤0.001

*Note.* Compared with before treatment, ^*∗*^*P* < 0.05; compared with single drug group, ^#^*P* < 0.05.

**Table 3:** Comparison of the levels of vascular endothelial cell injury markers in the two groups ($\bar{x}\pm s$).

Group	Number of cases	ET-1 (*μ*g/L)		NO (*μ*mol/L)	
		Before treatment	After treatment	Before treatment	After treatment
Single drug group	48	74.58 ± 10.36	66.58 ± 6.48^*∗*^	46.58 ± 7.84	52.78 ± 6.29^*∗*^
Joint group	48	75.74 ± 8.97	54.02 ± 5.17^*∗*#^	46.61 ± 8.05	61.77 ± 7.25^*∗*#^
*t*		0.586	10.497	0.018	6.489
*P*		0.279	≤0.001	0.493	≤0.001

*Note.* Compared with before treatment, ^*∗*^*P* < 0.05; compared with single drug group, ^#^*P* < 0.05.

**Table 4:** Comparison of adverse reactions between the two groups (*n* (%)).

Group	Number of cases	Gastrointestinal reaction	Flush	Dry mouth	Total
Single drug group	48	2 (4.17)	1 (2.08)	1 (2.08)	4 (8.33)
Joint group	48	1 (2.08)	2 (4.17)	0 (0.00)	3 (6.25)
*χ* ^2^					0.154
*P*					0.695

**Table 5:** Comparison of pregnancy outcomes between the two groups (*n* (%)).

Group	Number of cases	Cesarean section	Abnormal fetal heart rate	Neonatal asphyxia	Premature delivery	Stillbirth
Single drug group	48	17 (35.42)	8 (16.67)	7 (14.58)	6 (12.50)	1 (2.08)
Joint group	48	8 (16.67)^*∗*^	2 (4.17)^*∗*^	3 (6.25)	2 (4.17)	0 (0.00)
*χ* ^2^		4.381	4.019	1.786	2.182	1.011
*P*		0.036	0.045	0.181	0.140	0.315

*Note*. Compared with the single drug group, ^*∗*^*P* < 0.05.

## Data Availability

The data used to support the findings of this study are available from the corresponding author upon request.

## References

[1] Bakouei F., Delavar M. A., Mashayekh-Amiri S., Esmailzadeh S., Taheri Z. (2020). Efficacy of n-3 fatty acids supplementation on the prevention of pregnancy induced-hypertension or preeclampsia: a systematic review and meta-analysis. *Taiwanese Journal of Obstetrics & Gynecology*.

[2] Birukov A., Herse F., Nielsen J. H. (2020). Blood pressure and angiogenic markers in pregnancy. *Hypertension*.

[3] Tooher J., Thornton C., Makris A., Ogle R., Korda A., Hennessy A. (2017). All hypertensive disorders of pregnancy increase the risk of future cardiovascular disease. *Hypertension*.

[4] Van Winden K. R., Bearden A., Kono N. (2020). Low bioactive vitamin D is associated with pregnancy-induced hypertension in a cohort of pregnant HIV-infected women sampled over a 23-year period. *American Journal of Perinatology*.

[5] Oyagbemi A. A., Omobowale T. O., Ola-Davies O. E. (2018). Quercetin attenuates hypertension induced by sodium fluoride via reduction in oxidative stress and modulation of HSP 70/ERK/PPAR*γ* signaling pathways. *BioFactors*.

[6] Hamed S., Behnes M., Pauly D. (2018). Pentraxin-3 predicts short- and mid-term mortality in patients with sepsis and septic shock during intensive care treatment. *Clinical Laboratory*.

[7] Wei J., Wu Q. J., Zhang T. N. (2016). Complications in multiple gestation pregnancy: a cross-sectional study of ten maternal-fetal medicine centers in China. *Oncotarget*.

[8] Liu Z., Lang L., Li L., Zhao Y., Shi L. (2021). Evolutionary game analysis on the recycling strategy of household medical device enterprises under government dynamic rewards and punishments. *Mathematical Biosciences and Engineering : MBE*.

[9] Lai W. F., Wong W. T. (2021). Property-tuneable microgels fabricated by using flow-focusing microfluidic geometry for bioactive agent delivery. *Pharmaceutics*.

[10] Zhang Z., Cui F., Cao C., Wang Q., Zou Q. (2022). Single-cell RNA analysis reveals the potential risk of organ-specific cell types vulnerable to SARS-CoV-2 infections. *Computers in Biology and Medicine*.

[11] Marcinko D., Jakovljević M., Jakovljevic M., Jaksic N., Bjedov S., Mindoljevic Drakulic A. (2020). The importance of psychodynamic approach during COVID-19 pandemic. *Psychiatria Danubina*.

[12] Bener A., E Dafeeah E., Dafeeah E. E., Abou-Saleh M. T., Bhugra D., Ventriglio A. (2020). Co-morbidity between major depression and schizophrenia: prevalence and clinical characteristics. *Psychiatria Danubina*.

